# Evaluation Method of Human Resource Management Efficiency of Chain Retail Enterprises Based on Distributed Database

This article has been retracted.

**DOI:** 10.1155/2022/1860426

**Published:** 2022-02-01

**Authors:** Xiaolong Jiang, Mishal Sohail

**Affiliations:** ^1^Guangdong Mechanical & Electrical Polytechnic, Faculty of Logistics, Guangzhou 510515, China; ^2^Department of Computer Science, Superior University lahore, Pakistan

## Abstract

The calculation of human resource management efficiency evaluation method is large, which affects the technical efficiency and scale efficiency of evaluation results. Based on distributed database, an evaluation method of human resource management efficiency of chain retail enterprises is proposed. Genetic algorithm is applied to the design of distributed database to realize the best data allocation scheme. The distributed database is used to store the human resource information of chain retail enterprises to ensure the data consistency and information availability. Select the input and output elements that can best reflect the human resource management status of chain retail enterprises in the distributed database, design the management efficiency evaluation index system, and construct the DEA evaluation model. After testing, the technical efficiency and scale efficiency of the design method in this paper are higher than the evaluation methods of human resource management efficiency of chain retail enterprises based on principal component analysis and fuzzy comprehensive evaluation, which is conducive to management decision-making.

## 1. Introduction

Human resources were limited in the twenty-first century. Simultaneously, as a new capital, it has garnered increasing attention from society. Human resources may infuse organizations with life and help them compete more effectively. It is a term that refers to the efficient and rational deployment of this finite resource via materialization in order to optimize resource usage and economic advantages. Within an organization, good management enables the subjective initiative to flourish, operational costs to be reduced, and core competitiveness to be enhanced [1]. Level and efficiency have a direct impact on short-term progress and are critical in achieving long-term strategic goals. As a result, all sectors of society should manage their internal human resources scientifically and prudently in order to optimize revenues and foster long-term company growth [2]. However, as a result of the effect of factors such as inadequate professional quality and corporate culture on the managers of the majority of Chinese firms, the human resource management situation is often overlooked. For a long period of time, human resource management has been inefficient, and the realization of human resource value is not assured, which is very detrimental to long-term growth [3]. As a consequence, there is a pressing need to study management effectiveness.

A chain operation is a modern business idea that comprises of several stores selling similar goods and services. The transportation and service sectors are the most affected. Despite the fact that it has not developed in China for a long time, this new business model has changed the way traditional single-store operations are performed, accelerated product circulation, and simplified people's lives. It has steadily evolved into the primary organizational structure for China's commercial operations, demonstrating a high level of vitality and growth potential. At the moment, chain operation is prevalent in all retail formats for store sales in China and has evolved into the primary growth method employed by retail firms. The share of merchants engaging in chain operations is likewise expanding in the retail business. By and large, China's chain retailing business began late. Its management idea, technology application, human resource management level, and capital application are significantly inferior to those of worldwide chain organizations. The operating and management levels are still in their infancy. Human capital, as the basic driving force and critical element in the operation and growth of chain retail organizations, is not only the foundation of firm competitiveness, but also a critical component in achieving a competitive advantage and the primary driver behind profit creation. With rising competition from local and international chain retail organizations, Chinese businesses must prioritize human resources as their most precious asset, strive to improve human resource management efficiency, and then propel the retail sector forward. As a result, this study provides a distributed database-based assessment approach for chain retail firms' human resource management efficiency, which shows the current condition, assists enterprises in optimizing resource allocation, and enhances their market competitiveness.

## 2. Evaluation Method of Human Resource Management Efficiency of Chain Retail Enterprises Based on Distributed Database

### 2.1. Design of Distributed Database Based on Genetic Algorithm

Different from centralized database management system, distributed database involves data distribution, joint query of multiple data sets, and so on. In order to improve the performance of human resource management in chain retail enterprises in data processing, it is necessary to design distributed database. Data dissemination is a critical phase in the development of a distributed database [4]. The following mathematical definition may be used to describe data distribution: The system consists of multiple data stations that are linked through a network. The program transaction set is network-based. A data set serves as the foundation for program transaction activity. Then, the data allocation algorithm must address the following problem: design an algorithm, reasonably configure the copies of the data set across multiple sites in order to maximize the overall performance of the system while minimizing total cost, and record the scheme as the best allocation scheme at the time. For the purpose of conducting research on the optimal data allocation algorithm, the current algorithms primarily include a grouping local optimization algorithm aimed at minimizing the cost of data fragment storage, a clustering optimization algorithm based on calculating the minimum average value, a vertical fragment clustering method based on attribute correlation degree, and a clustering and allocation algorithm combined. While each of the preceding techniques has its own set of pros and downsides, the optimization result obtained by combining clustering and allocation is the best. However, since each data unit must be processed individually, the algorithm process is complicated, time-consuming, and in need of improvement. It presents a genetic algorithm-based technique for clustering data allocation. The concept is as follows: various data stations are grouped into distinct clusters depending on their communication costs with other stations. Following the clustering procedure, the genetic algorithm is employed to investigate the data unit allocation. Finally, the data allocation plan is selected using the minimal overall cost criteria. The cost of data processing and the cost of transmission between stations are the two basic components of determining the cost of communication between various stations. The total cost between stations is the sum of the two. At the same time, there are certain characteristics to the cost across places. First, the generating value has no direction; second, the communication cost between sites is directly proportional to their distance; third, the communication cost between sites is directly proportional to their distance. Allocating data units to distinct clusters performs better than assigning them to stations directly, which may increase station communication efficiency while lowering costs. After the site clustering process is completed, the communication cost between clusters and inside each cluster must be defined and clarified. If a single cluster contains multiple stations, the average communication cost can be defined as *α*_1_, and the calculation formula is as follows:

(1) $$\begin{array}{c} \alpha_{1}=\frac{\sum_{i=1}^{m}\beta \left(p_{i},p_{j}\right)}{m\left(m-1\right)}. \end{array}$$

In formula (1), *m* represents the number of transactions; *p* stands for station; *i*, *j* indicate serial number; *β* indicates the communication cost. The communication cost between different clusters can be defined as *α*_2_, and the calculation formula is as follows:

(2) $$\begin{array}{c} \alpha_{2}=\frac{\sum_{j=1}^{n}\sum_{i=1}^{m}\beta \left(p_{i},p_{j}\right)}{mn}. \end{array}$$

In formula (2), *n* represents the number of stations. The total communication cost of all clusters in the system can be defined as *α*_3_, and the calculation formula is as follows:

(3) $$\begin{array}{c} \alpha_{3}=\frac{\sum_{j=1}^{m}\sum_{i=1}^{m}\beta \left(p_{i},p_{j}\right)}{m^{2}}. \end{array}$$

The data optimum allocation based on genetic algorithm in the following stage is based on the prior definition and analysis of the internal communication cost of clusters and the communication cost between clusters. The processing procedure of the genetic algorithm is enhanced based on the application features of the data allocation method.  Figure 1 depicts the upgraded database's allocation processing flow.

The data allocation process based on genetic algorithm is based on the data structure, and the final data allocation scheme is obtained through the relevant operations of genetic algorithm.

### 2.2. Store Human Resource Information of Chain Retail Enterprises Based on Distributed Database

The data distribution method, which is based on a genetic algorithm, enables the storage to be processed optimally. It is utilized to store human resource information on this basis, hence increasing the model's operational efficiency. At the moment, chain retail firms' essential human resource management data is scattered across numerous data centers. Horizontal splitting is used in data centers to spread production data. The data nodes operate in the conventional minicomputer+storage+relational database manner, and data synchronization is accomplished by a replication server or data transfer [5]. Through replication definition and replication protocol, replication primarily utilizes Sybase's replication server technology to automatically synchronize the master node's data activities with the slave node database. Data transmission is mostly comprised of small batch file transmission and data warehousing in order to achieve full data synchronization, which is an asynchronous quasi-real-time synchronization approach [6]. To execute the transaction, the client navigates to the associated storage node using the transaction middleware in conjunction with the data fragmentation specification. For backup purposes, the core data node uses only the dual machine hot standby or active standby two-way replication approach. In the event of a failure, the changeover time is lengthy, and the danger of a single point of failure remains significant. As a result, it presents a paradigm for distributed consistent data storage and computation. The basic composition is shown in Figure 2.

As shown in Figure 2, the information data is stored in MySQL database, and multiple storage nodes ensure the consistency of data copies based on P1XOS like protocol [7]. The open source InnoDB is used as the data storage engine, and Zookeeper is used to implement the election component to realize the distributed consistent storage system. The functional modules of the storage node are shown in Figure 3.

As shown in Figure 3, each node includes five functional modules. The role control module is mainly built by Zookeeper client, an open-source distributed application coordination service. This module's purpose is to facilitate the election and recovery of leaders. The leader service module is composed of three modules: read requests, write requests, and proposer requests. The follower service module consists of three modules: read follower, follower recovery, and request service. The storage engine is InnoDB. The role control module is in charge of the leader service module, which includes the read request module, the write request module, and the proposer module. The role control module coordinates the follower service module and decides whether the leader should be elected or restored based on the node's operating condition at the moment. Because InnoDB enables acid transactions and four layers of transaction isolation, the storage engine module utilizes the InnoDB build port. It provides row-level locks and foreign key restrictions, which enables it to fulfill write concurrency needs. Generally, an InnoDB engine may be placed in a file space with no operating system-imposed limit on the table size, referred to as shared table space, and the same database can also be split over numerous files [8, 9]. It may also be stored in several independent table areas, each of which is limited in size by the operating system's file system. InnoDB uses technologies including adaptive hash indexing, preread, insert cache, and double write to improve performance, as well as a next key locking mechanism to prevent unreal reading. Memory pool technologies are used extensively in InnoDB, including the creation of a buffer pool, log cache, and additional memory pool. The buffer pool is responsible for the adaptive hash index and index page, as well as the database page, data dictionary information, insert cache page, lock information, and undo page. It is used to keep track of data needed by system processes or threads, as well as to create a fast read and write disk cache. The background thread is used by InnoDB to refresh the data in the memory pool. The refresh operation reads the data files into the InnoDB buffer pool page by page to guarantee that the buffer pool's memory cache can hold the most recent data [10, 11]. The updated data is cached using the least recently used (LRU) technique, refreshed on a regular basis, and written to the disk file as a modified data page. The client's queries will be sent to various nodes in distributed applications. Leader, follower, and learner are the cluster nodes. Data write proposals and data write operation requests must be proposed by the leader. Data read services and data write applications to the leader are handled by the follower. Accepting data write proposals and submitting write operations to the database are the responsibilities of the learner. In addition, the leader has a term of office, and the leader election may be held on a regular basis or manually intervened in as required [12]. In most cases, a fast leader selection method is utilized to elect leaders. The following properties are present in the node during election in the algorithm, as illustrated in Table 1.

After selecting the leader, the distributed system needs to synchronize data in the cluster to ensure the data consistency of all nodes. Data synchronization is divided into data synchronization and data write synchronization. The synchronization is based on the log. The transaction ID is used to identify all data operations performed by the node and is recorded to the log. As transit, the transaction ID may be captured. To begin, the follower sends a synchronization request to the leader. The request also contains the transmission of the company's most recent data operation. The leader will compare the follower to its transit to ascertain what data is missing and will provide the follower the missing operation report. Following receipt of the operation log, the follower will locally combine the logs in order to take action on the data. This ensures data consistency and improves the availability of information.

### 2.3. Design the Evaluation Index System of Human Resource Management Efficiency

Starting with the human resource management efficiency of chain retail enterprises, select the input and output elements that best reflect the human resource management status of chain retail enterprises, using the stored human resource management information and fully referring to the design principles of the index system, and design the evaluation index system.  Table 2 shows the evaluation index system.

The total amount of human resources refers to the total amount of human resources in the enterprise, which plays a basic role in promoting the operation and development of the enterprise in a certain period of time [13]. Although the number of workers will change over time as a result of external recruiting and as a result of resignations, dismissals, and other causes, the overall quantity of human resources in the organization will remain relatively steady over time. This study utilizes the total number of chain retail establishments in that year as the index's particular data. The human resource flow rate is defined as the ratio of the net difference between the inflow and outflow of enterprise human resources during a certain time period to the total number of workers over the preceding period. This indicator is intended to assess the enterprise's human resource team's stability [14]. A high turnover rate of human resources is an unavoidable byproduct of today's more tough market rivalry. Employees may discover their own advantages and the finest work content in fast-paced work environments, as well as obtain the best person-postmatch by changing their jobs [15]. However, when the flow of human resources surpasses a specific threshold, it shows that there are issues with the enterprise's incentive structure or corporate culture. At this point, the firm must assess its existing status and make necessary adjustments. Enterprises should not overemphasize personnel stability and excessively restrict talent flow during the development process but should instead maintain an appropriate flow of personnel, which will not only contribute to the development of the enterprise but will also promote free and benign competition among enterprises, which is a necessary condition for the optimal allocation of human resources [16]. The calculation formula of human resource turnover rate is as follows:

(4) $$\begin{array}{c} \omega =\frac{N_{1}-N_{2}}{N_{2}}. \end{array}$$

In formula (4), *ω* represents the turnover rate of human resources; *N*_1_ represents the total number of employees in the current period; *N*_2_ represents the total number of employees in the previous period. The proportion of senior executives refers to the proportion of senior executives in all employees of the enterprise. This indicator captures the organization's management capability and efficiency in a single dimension. To a certain degree, the presence of more senior executives implies that the greater the enterprise's size, the quicker its growth, and vice versa. Because marketing professionals account for more than half of all workers, they play a critical role in corporate growth and are a critical source of competitiveness for businesses [17]. The educational structure may indicate the average degree of education of workers, with the average number of years of education serving as the statistical indicator. According to educational levels, human resources can be classified as personnel with a doctorate, personnel with a master's degree, personnel with a bachelor's degree, and personnel with a college degree or less. The average years of education at each educational level are 22.5, 18.5, 16, and 15 years, respectively [18–20]. The average length of education of employees can be calculated by the following formula:

(5) $$\begin{array}{c} \vartheta =\sum \varphi \bar{M}. \end{array}$$

In formula (5), *ϑ* represents the average education years of employees; *φ* represents the proportion of employees in this education stage; $\bar{M}$ means the average years of education at this stage. Age structure refers to the average age of employees in the enterprise, reflecting the younger level of the enterprise. The age structure of human resources can be divided into three stages: personnel under the age of 35, personnel aged 36-45, and personnel over the age of 46. The average ages of the three age groups were 30.5, 40.5, and 50.5 years, respectively. The age structure of enterprise human resources can reflect the aging level of the enterprise, the innovation degree of employees, the personnel development strategy of the enterprise, and many other aspects [20]. These factors will have a certain impact on the enthusiasm and creativity of employees and even the strategic execution of the organization. The specific calculation formula of the index is as follows:

(6) $$\begin{array}{c} \eta =\sum \varphi \bar{Y}. \end{array}$$

In formula (6), *η* represents the average age of employees; $\bar{Y}$ represents the average age of this age group. The title structure can reflect the degree of specialization of an enterprise's personnel and represent the ability level of employees to use professional skills to solve various resource problems in their work. The human resource professional title level is divided into three levels: senior, intermediate, and primary professional title. The three levels are assigned with 3, 2, and 1 points, respectively. The proportion of the distribution of each professional title segment of employees is multiplied by the corresponding score of the professional title stage to obtain the professional title level of employees by weighted average.

### 2.4. Establish the Efficiency Evaluation Model of Human Resource Management

The methods used by scholars at home and abroad to evaluate the efficiency of human resource management primarily include principal component analysis, fuzzy comprehensive evaluation, data envelopment analysis, subjective and objective workload evaluation, genetic algorithm-based model solution, ranking method approaching ideal solution, and questionnaire survey method. Each of the strategies listed above has its own set of requirements. In light of the industry's unique characteristics in terms of business and environment, the DEA method's benefits include high accuracy, the absence of the requirement to preset the function form, and an easy-to-use operation procedure. It is capable of assessing the human resource management practices of chain retail organizations. As a result, this study will use the DEA approach to develop an assessment model of chain retail firms' human resource management efficiency. The DEA model is classified as input- or output-oriented. When a DEA model is used to do real calculations, the guidance type should be chosen based on the current scenario and the complexity of the input or output. The application steps are shown in Figure 4.

The use of DEA should primarily follow the aforementioned fundamental processes, as shown in Figure 4, from the definition of assessment goals through the formulation of countermeasures and proposals, therefore establishing a closed-circuit circulation system. DEA is not required to predefine a certain input-output production function form. As a result, the DEA method's calculating procedure is very straightforward and has a broader applicability range. It is capable of assessing the effectiveness of complicated and dynamic decision-making units and mitigating the effects of inappropriate function assignment. The DEA method ignores the logical relationship between indicators and does away with the need to preset indicator weights. Its weight is computed at the same time as the indicator data, removing the volatility caused by subjectivity in assignment. The DEA methodology does not need normalizing the data units of each index when measuring the efficiency of a decision-making unit; instead, it may keep the difference between each data unit, greatly simplifying the method's operation. The output index does not correspond to the input indicators when the DEA is used as the foundation for the first mock test. This drives us to enhance output indicators and use the model to quickly evaluate relative effective efficiency. Difference, efficiency, and sensitivity studies may all be performed using the DEA method. We can completely comprehend resource use in each decision-making unit in order to make right and accept resource allocation judgments at a later stage. The scale of the same type of the same firm in the same era is the first BCC mock test. This paper selects this model to evaluate the efficiency of the chain retail enterprises' human resource management. The constructed evaluation model is as follows:

(7) $$\begin{array}{c} \left\{\begin{array}{c} \min\lambda =\lambda^{+},\\ \overset{u}{\underset{y=1}{\sum }}a_{xy}\gamma_{y}+\kappa^{-}=\lambda a_{xy},\\ \overset{u}{\underset{y=1}{\sum }}b_{hy}\gamma_{y}-\kappa^{+}=b_{hy},\\ \overset{u}{\underset{y=1}{\sum }}\gamma_{y}=1. \end{array}\right. \end{array}$$

In formula (7), *λ* represents the input proportional variable; *λ*^+^ represents the input surplus; *a*_*xy*_ and *b*_*hy*_ represent the *x* input index data and *h* output index data of decision-making unit *y*, respectively; *γ*_*y*_ represents linear combination coefficient; *u* represents the number of decision-making units; *κ*^+^ and *κ*^−^ represent residual and relaxation variables. If *λ*^+^ = 1, the DMU is DEA weakly efficient. If *λ*^+^ = 1 and *κ*^+^ = *κ*^−^, the DMU is DEA valid. If 0 < *λ*^+^ < 1, the DMU is DEA and invalid. In the process of evaluating the human resource management efficiency of chain retail enterprises, it is not easy when *κ*^+^ = *κ*^−^. Therefore, by introducing Archimedean infinitesimal *ε*, the following model can be obtained:

(8) $$\begin{array}{c} \min\left[\lambda -\varepsilon \left(e^{T}\kappa^{-}+e^{T}\kappa^{+}\right)\right]=\lambda^{+}. \end{array}$$

In formula (8), *e*^*T*^ represents the transpose matrix of natural constants. At this time, when the scale efficiency is equal to 1, it indicates that the decision-making unit is effective. When the scale efficiency is less than 1, it indicates that the decision-making unit is not effective and is not in the best production frontier. So far, the construction of human resource management efficiency evaluation model of chain retail enterprises has been completed.

## 3. Experiment

### 3.1. Experimental Preparation

This experiment selects 30 chain retail enterprises as the research sample, including 6 listed companies and 8 Sino foreign joint ventures. Therefore, the selection of samples is representative and comprehensive, which not only facilitates the data operation but also accurately evaluates the human resource management efficiency of chain retail enterprises. This paper will select the data of these 30 chain retail enterprises from 2016 to 2020 for research. The Deap2.1 software is used to perform data envelopment analysis on the input-output index data of each decision-making unit to determine the human resource management efficiency of chain retail firms from 2016 to 2020, using the aforementioned sample enterprises as 30 decision-making units.

### 3.2. Experimental Results and Analysis

In order to verify the effectiveness of the evaluation method proposed in this paper, it is compared with the evaluation methods of human resource management efficiency of chain retail enterprises based on principal component analysis and fuzzy comprehensive evaluation. The technical efficiency and scale efficiency are selected as the evaluation indexes to verify the evaluation effect of each method. The experimental results are shown in Tables 3 and 4, respectively.

The average technical efficiency of the design method in this paper is 0.947, which is 0.226 and 0.128 higher than the evaluation methods of human resource management efficiency of chain retail enterprises based on principal component analysis and fuzzy comprehensive evaluation, respectively, as shown in Table 3. The average scale efficiency of the design method in this paper is 0.961, which is 0.208 and 0.139 higher than the evaluation methods of human resource management efficiency of chain retail enterprises based on principal component analysis and fuzzy comprehensive evaluation, respectively, according to the results in Table 4. As a result, the design process may enhance technical and scale efficiency, satisfy the application needs of real businesses, assist businesses in making management choices, and optimize structure, resulting in increased revenue and value.

## 4. Conclusion

In terms of investment, the evaluation indicators are selected from two aspects: human resource scale and human resource structure. In terms of output, indicators are selected from three aspects: profitability, business growth ability, and development innovation ability to form an innovative evaluation index system. The construction of the index system has laid a solid foundation for the follow-up research of this paper. This study is a new perspective on the efficiency of chain retail enterprises and provides a theoretical reference for the allocation. However, this paper has not been perfectly presented in the process of text description or empirical analysis, which needs to be improved by the latecomers. In order to fully understand the efficiency, it is necessary to establish an index system covering enterprise strategy, performance management, salary management, organizational structure, and so on, so as to minimize the subjectivity of index selection. There is a time difference between the input and output of any resource, and there is still no answer to the determination of the lag period of the output of human resource allocation. This paper does not consider the lag problem in the research, which is another deficiency of this paper. Future research should pay attention to the determination of lag length to make the research closer to reality.

## Figures and Tables

**Figure 1:** Database allocation processing flow.

**Figure 2:** Basic composition of information node.

**Figure 3:** Functional modules of storage node.

**Figure 4:** Application steps of DEA.

**Table 1:** Node attribute list.

Node	Meaning	Explain
Node Id	Node ID number	It needs to be specified manually in the configuration file
View	Status of all nodes after each election	The initial value is 0, and the view will increase by 1 after each election
Trans	Proposal transaction serial number	The initial value is 0, and trans will increase by 1 after each proposal is passed
Clock	Election count for service	Initial 0
State	Voter status	Node state set

**Table 2:** Evaluation index system of human resource management efficiency.

Primary index	Secondary index	Tertiary indicators
Investment	Human resource scale	Total human resources
		Turnover rate of human resources
		Proportion of senior executives
		Proportion of marketing personnel
	Human resource structure	Educational structure
		Age structure
		Title structure
Produce	Profitability	Net profit at the end of the year
	Business growth ability	Net profit growth rate
		Growth rate of total assets
	Develop innovation ability	Proportion of handling fees and commissions
		Return on net assets

**Table 3:** Comparison results of technical efficiency.

Year	The method of this paper	Method based on principal component analysis	Method based on fuzzy comprehensive evaluation
2016	0.952	0.726	0.828
2017	0.946	0.711	0.814
2018	0.962	0.718	0.802
2019	0.925	0.705	0.816
2020	0.948	0.748	0.836

**Table 4:** Comparison results of scale efficiency.

Year	The method of this paper	Method based on principal component analysis	Method based on fuzzy comprehensive evaluation
2016	0.962	0.756	0.825
2017	0.958	0.748	0.836
2018	0.964	0.762	0.817
2019	0.957	0.751	0.808
2020	0.961	0.749	0.823

## Data Availability

Data are available on request.

## References

[1] Pepitone J. S. (2019). Are you considering evidence-based human resource management decision-making?. *Management Services*.

[2] Guiyao T., Lin C., Yang C., Songbo L. (2019). Commitment to human resource management of top management team, green human resource management and firm performance: the moderating effect of firm size. *Nankai Business Review*.

[3] Juan W. A. N. G., Zhe Z. H. A. N. G., Ming J. I. A. (2019). The research on the relationship between socially responsible human resource management and counterproductive work behavior: a moderated mediation model. *Journal of Industrial Engineering and Engineering Management*.

[4] Muzammal M., Qu Q., Nasrulin B. (2019). Renovating blockchain with distributed databases: an open source system. *Future Generation Computer Systems*.

[5] Lotfi N. (2019). Data allocation in distributed database systems: a novel hybrid method based on differential evolution and variable neighborhood search. *SN Applied Sciences*.

[6] Khamis A. D., Subair S. (2019). Security framework for distributed database system. *Journal of Data Analysis & Information Processing*.

[7] Schuler R., Kesselman C. (2020). Chisel: a user-oriented framework for simplifing database evolution. *Distributed and Parallel Databases*.

[8] O'Leary D. E. (2019). Some issues in blockchain for accounting and the supply chain, with an application of distributed databases to virtual organizations. *Intelligent Systems in Accounting, Finance and Management*.

[9] Klbe S., Sattler K. U., Baumann S. (2021). Patchindex: exploiting approximate constraints in distributed databases. *Distributed and Parallel Databases*.

[10] Man-man C. A. O., Mian W. A. N. G. (2019). Research on accurate classification and simulation of distributed databases. *Computer Simulation*.

[11] Chauhan N. R., Tripathi S. P. (2021). Optimal admission control policy based on memetic algorithm in distributed real time database system. *Wireless Personal Communications*.

[12] Qaosar M., Zaman A., Siddique M. (2019). Privacy-preserving secure computation of skyline query in distributed multi-party databases. *Information*.

[13] Gurmu A. T., Ongkowijoyo C. S. (2020). Predicting construction labor productivity based on implementation levels of human resource management practices. *Journal of Construction Engineering and Management*.

[14] Za A., Mfo B., Hk C. (2020). Does servant leadership moderate the link between strategic human resource management on rule breaking and job satisfaction?. *European Research on Management and Business Economics*.

[15] Jia H., Lijuan X., Huan J. (2019). Development of indexes for evaluating nursing human resource efficiency in geriatric department based on data envelopment analysis. *Journal of Nursing Science*.

[16] Yanling W. E. N. G., Lihui C. H. E. N. G., Yamei B. A. I., Yulei S. O. N. G. (2019). Construction of evaluation index system of nursing human resources efficiency. *Chinese Nursing Research*.

[17] Ahammad M. F., Glaister K. W., Gomes E. (2020). Strategic agility and human resource management. *Human Resource Management Review*.

[18] Anlesinya A., Susomrith P. (2020). Sustainable human resource management: a systematic review of a developing field. *Journal of Global Responsibility*.

[19] Khan S. I., Bartram T., Cavanagh J., Hossain M. S., Akter S. (2019). 'Decent work' in the ready-made garment sector in Bangladesh: the role for ethical human resource management, trade unions and situated moral agency. *Personnel Review*.

[20] Cooper B., Wang J., Bartram T., Fang L. C. (2019). Well-being-oriented human resource management practices and employee performance in the Chinese banking sector: the role of social climate and resilience. *Human Resource Management*.

